The article "A Novel Approach to Classifying Breast Cancer Histopathology Biopsy Images Using Bilateral Knowledge Distillation and Label Smoothing Regularization" was retracted in 2023. Reasons: signs of a paper mill; compromised peer review; unreliable results or conclusions.

# A Novel Approach to Classifying Breast Cancer Histopathology Biopsy Images Using Bilateral Knowledge Distillation and Label Smoothing Regularization

**DOI:** 10.1155/2021/4019358

**Published:** 2021-10-20

**Authors:** Sushovan Chaudhury, Nilesh Shelke, Kartik Sau, B. Prasanalakshmi, Mohammad Shabaz

**Affiliations:** ^1^University of Engineering and Management, Kolkata, India; ^2^Priyadarshini Indira Gandhi College of Engineering, Nagpur, India; ^3^Department of Computer Science, King Khalid University, Abha, Saudi Arabia; ^4^Arba Minch University, Ethiopia

## Abstract

Breast cancer is the most common invasive cancer in women and the second main cause of cancer death in females, which can be classified benign or malignant. Research and prevention on breast cancer have attracted more concern of researchers in recent years. On the other hand, the development of data mining methods provides an effective way to extract more useful information from complex databases, and some prediction, classification, and clustering can be made according to the extracted information. The generic notion of knowledge distillation is that a network of higher capacity acts as a teacher and a network of lower capacity acts as a student. There are different pipelines of knowledge distillation known. However, previous work on knowledge distillation using label smoothing regularization produces experiments and results that break this general notion and prove that knowledge distillation also works when a student model distils a teacher model, i.e., reverse knowledge distillation. Not only this, but it is also proved that a poorly trained teacher model trains a student model to reach equivalent results. Building on the ideas from those works, we propose a novel bilateral knowledge distillation regime that enables multiple interactions between teacher and student models, i.e., teaching and distilling each other, eventually improving each other's performance and evaluating our results on BACH histopathology image dataset on breast cancer. The pretrained ResNeXt29 and MobileNetV2 models which are already tested on ImageNet dataset are used for “transfer learning” in our dataset, and we obtain a final accuracy of more than 96% using this novel approach of bilateral KD.

## 1. Introduction

Breast cancer is the most lethal type of tumour in women worldwide, second only to lung cancer in terms of prevalence. In the most common type of breast cancer, which is popularly known as invasive ductal carcinoma (IDC), the cancer develops in the milk ducts of the breast and then rapidly spreads to involve the surrounding structures. Invasive ductal carcinoma is so progressive that it can even infiltrate the lymph nodes and the circulatory system, which leads to the cancer spreading to various parts of the body. Even though invasive or infiltrating ductal carcinoma may be rapidly progressive, but it is still a treatable condition at least when identified in its initial stages [1]. Machine learning is a branch of artificial intelligence that employs a variety of statistical, probabilistic, and optimization techniques that allow computers to “learn” from past examples and to detect hard-to-discern patterns from large, noisy, or complex datasets. As a result, machine learning is frequently used in cancer diagnosis and detection. Machine learning and deep learning approaches may help radiologists to a large extent by helping to detect breast cancer at an early stage by identifying useful patterns in malignant cells. The learnt patterns can be used to classify the unknown images of the breast as benign or malignant. Mammography, ultrasonography, and histological biopsies are some of the numerous options for BCD. Mammograms can help to understand calcification in human breast, whereas studying histology images remains a challenge due to its complexity in pattern identification. This study analyzes the gene activities of the survival vs. deceased for each therapy, and the potential biomarkers will help to identify the best therapy for the patients based on their gene expression test. This model has very high accuracy levels, and it uses a hierarchical model as a tree that includes one-versus-rest classifications. In 2012, there were roughly 1.7 million new cancer cases (representing 25% of all malignancies in women) and 0.5 million cancer deaths (representing 15% of all cancer fatalities in women). In 140 nations, ductal carcinoma is the most prevalent cancer diagnosis among females, and it is the primary cause of cancer death in 101 nations. According to McGuire [2], histological study of breast cancers can also reveal the stage of the disease or the extent to which the cancer has spread. This is measured in two ways: by the size of the tumour and by assessing the involvement of regional lymph nodes. Both of these variables provide valuable prognostic data for patient care. Smith et al. [3] recommend screening practices for the early recognition of breast cancer. Computer-aided diagnosis of ductal carcinoma can advance the performance of radiologists in several folds as explained by Filipczuk et al. and Kowal et al. [4, 5]. The simple idea of the CAD system is to take raw descriptions from different modalities like mammogram and histology images and preprocess them. This preprocessing includes amending size, contrast, and brightness and performing augmentation in case input data which are scarce. The next step involves segmentation to critically identify the regions of interest in the image so that the system only learns the relevant part of the image and not the noise part. The third stage is to extract features from a region of interest (ROI), which is usually done using CNN, which handles automatic feature extraction by producing feature maps at each convolution layer and regularising the models with dropouts so that they do not fit [6]. The higher-order feature maps are flattened, and classification is performed using the class probabilities generated by a softmax layer. These models, however, are massive, containing millions (if not billions) of parameters, and so cannot be used on edge devices. The technique is being tested on the BACH dataset, a large histology dataset for breast cancer detection, to reduce computational complexity. The concept is to represent compression by having a larger and more sophisticated pretrained network that teaches a smaller network (students) step by step (teacher). Indeed, the theoretical search space for more complicated models is bigger than that of a smaller system [7, 8]. However, if we suppose that the equivalent (or even comparative) convergence can be attained using a smaller link, then the convergence space of the teacher system should connect with the solution space of the student system. Tragically, that by itself does not ensure union of the solution space for the student network and the teacher network in a similar area. The convergence of the student network may be completely different from the convergence of the teacher network [9].

The basic steps of knowledge distillation are given as follows.

1. Train the teacher network: The complex teacher network is first trained using the whole dataset on high-performing GPUs
2. Establish a link of correspondence: The student network is then designed and a correspondence needs to be formed between each output of the simple student network and the complex teacher network
3. Forward propagation of knowledge through the teacher network: Feedforward data through the teacher network to get all intermediate outputs; apply augmentation (if any) to the same
4. Backpropagation through the student network: The output from the teacher and the correspondence relation are used to backpropagate the error to the student. Therefore, the student network learns to imitate the “knowledge” of the teacher

## 2. Related Work

Koboldt et al. [10] studied key ductal carcinoma by genomic DNA copy arrays, DNA methylation, exome sequencing, messenger RNA arrays, micro-RNA sequencing, and opposite-segment protein arrays. The different classifications of breast cancers are researched in accordance with WHO standards [11]. They outline the methods required to examine the histological description of breast cancer, similar to the one explained by Veta et al. [12]. With the introduction of whole slide imaging (WSI) scanners, which can be affordable and high-throughput histopathology slide digitalization, this study topic has become particularly relevant, with the goal of substituting the optical microscope as the principal tool used by pathologists. Breast cancer classification from histological photos is of considerable therapeutic value, according to [13], although it is yet to be studied. The multiple classification of ductal carcinoma has a purpose to find the subcategories of breast cancer (ductal carcinoma, fibroadenoma, lobular carcinoma, etc.). However, multiclassification of breast cancer from histopathology pictures faces 2 major challenges: (1) sorting of binary classes (benign and malignant) and (2) minor variances in various classes due to the wide diversity of high-resolution picture appearances, strong coherency of malignant cells, and large colour distribution inhomogeneity. As per Sharma et al. [14], special attention was given to histopathology images in the BACH dataset. A model of careful consideration was proposed where the network emphasizes learning from patches and records good accuracy in multilevel classification. Kausar et al. [15] experimented with a number of deep convolutional models, using colour normalisation as a normalisation strategy before applying augmentation to the input data. Praveena Anjelin and Ganesh Kumar [16] experimented with different transfer learning techniques and pretrained models such as MobileNetV2, AlexNet, ResNet, and VGGNet on the BACH dataset. Several efforts in the subject of knowledge distillation have also been completed. Ba and Caruana [17] investigated with the CIFAR10 dataset and detected that a large network is capable of training smaller networks in patches that are quite shallow but are capable to match the accuracy of deep neural nets, and since they need not be necessarily deep, the computational complexity can be reduced. Hinton et al. [18] found startling findings on MNIST, demonstrating that condensing the knowledge from an ensemble of models into a single model can greatly improve the acoustic model of a widely used commercial system [19]. Often the finest outcomes are attained by assembling millions of individual classifiers, which is a computationally expensive task. In [20], researchers offer a strategy for “compressing” big, complicated ensembles into smaller, quicker models with little to no performance loss. Dipalma et al. [21] utilised knowledge distillation with model compression to address challenging problems in whole slide images, such as histology. Knowledge distillation has been used in object detection by Dai et al. [22], face recognition by Ge et al. [23], semantic segmentation by He et al. [24], classification of chest X-ray abnormalities by Ho and Gwak [25], and to regain land surface temperature from MODIS daytime mid-infrared data by Tang and Wang [26]. Knowledge distillation was used to enhance the computational efficiency of breast cancer diagnosis by Garg et al. and Thiagarajan et al. [27, 28]. They stress that in a variety of applications, such as medical image analysis, weakly supervised instance labelling utilising simple picture-level labels rather than costly fine-grained pixel annotations are critical. In contrast to traditional computer vision instance segmentation, the challenges we address are characterised by a small number of training photos and nonlocal patterns that lead to diagnosis. Motivated by all of these KD applications, as well as the use of KD and computationally efficient neural nets for training large WSI as in BACH images of the breast, we decided to focus on bilateral knowledge distillation, in which the teacher and student learn from each other and improve each other's performance, as shown in [29–31].

## 3. Methodology

### 3.1. Dataset and Preprocessing

For our experiments, we used ICIAR 2018 Grand Challenge on Breast Cancer Histology dataset [32] as described in Figure 1. The dataset is comprised of haematoxylin and eosin (H&E) stained breast microscopic anatomy research and whole slide images labelled as traditional, benign, in-place cancer, or invasive cancer. The clarification was performed by 2 clinical specialists and images with conflict were disposed of. A total of 400 microscope images are in the collection, out of which 100 each are normal images, benign images, in situ carcinoma, and invasive carcinoma. All microscopy images are on.tiff format, and their specifications are given below in Table 1.

The BACH dataset comprises of about 400 histological microscopic images of the breast stained with haematoxylin and eosin (H&E). Conferring to the major cancer type in each image, these photos are categorized as [N] normal, [B] benign, [I] in situ carcinoma, or invasive carcinoma, with 100 labels each. The dataset was distributed into 70 : 30 train-test subgroups for the studies we ran. Because of the variances in staining methods, scanner colour response, and tissue preparation, the staining process is a complex process that might result in undesired colour variations among tissue types. We employ a technique called structure-preserving colour normalisation with sparse strain separation since colour variance across pictures can affect performance. The approach uses one picture as the target, and the other images are normalised by merging their separate stain density maps with the target image's stain colour base, maintaining the morphology. After that, the modified dataset is scaled between 0 and 1, and each channel is normalised to the ImageNet dataset. ImageNet project is a large visual database used in visual object recognition in software research and is tested and trained on more than 14 million images of various types, both labelled and unlabelled. We use online data augmentation techniques to provide variety to the training dataset, allowing the network to generalise to new datasets. Because the histological pictures are rotationally invariant, horizontal and vertical flips with rotations ranging from -25 to 25 degrees were also included. As augmentation methods, random zoom and intensity shifts were also utilised.

### 3.2. Knowledge Distillation in Theory

Knowledge distillation refers to distilling facts from a complex teacher model into a relatively weak and light student model. However, it is can be better summarized as a label smoothing regularization technique. The outcome of knowledge distillation depends not only on the similarity information between teacher categories but also on the regularization of soft goals. The softening regularization of the label refers to the model training by the exchange of one hot label and soft smoothed label between the teacher and the student. Loss function of label smoothing regularization (LSR) for a network *S* is as follows. For every training instance *x*, *S* outputs the probability of each label as shown in the following equation:

(1) $$\begin{array}{c} a\in \left\{1..A\right\}\text{: }r\left(a\left|y\right.\right)=\text{soft}\max\left(T_{a}\right)=\frac{\exp\left(T_{a}\right)}{\sum_{f-1}^{A}\left(T_{f}\right)}, \end{array}$$

where *S* is a neural network to train, *T*_*f*_ is the logit of the neural network, and *S* is given in the following equation.

(2) $$\begin{array}{c} n^{\prime }\left(a\right)=\left(1-\beta \right)n\left(a\right)+\beta v\left(a\right), \end{array}$$

where *n*′(*a*) is the smoothed labelled distribution, is a mixture of *n*(*a*), and is a fixed distribution *v*(*a*) with weight *β*. Now, *v*(*a*) is uniform distribution as *v*(*a*) = [1/*A*].

The smoothed entropy loss *B*(*n*′, *r*) is defined over the smoothed label as in the following equation.

(3) $$\begin{array}{c} B\left(n^{\prime },r\right)=-\overset{A}{\underset{f-1}{\sum }}n^{\prime }\left(a\right)\log r\left(a\right)=\left(1-\beta \right)B\left(n,r\right)+\beta B\left(v,r\right)=\left(1-\beta \right)B\left(n,r\right)+\beta \left(C_{\text{AM}}\left(v,r\right)+B\left(v\right)\right), \end{array}$$

where *C*_AM_ is the Kullback-Leibler divergence and *C*(*a*) denotes the entropy of *v* and is a constant for the fixed uniform distribution *v*(*a*).

The loss function for label smoothing of neural network *S* can be written as in the following equations:

(4) $$\begin{array}{c} M_{\text{MO}}=\left(1-\beta \right)B\left(n,r\right)+\beta C_{\text{AM}}\left(v,r\right), \end{array}$$

(5) $$\begin{array}{c} m_{\text{AC}}=\left(1-\beta \right)B\left(n,r\right)+\beta C_{\text{AM}}\left(r_{\pi }^{x},r_{\pi }\right), \end{array}$$

where *B*(*n*, *r*) is the minimized cross-entropy and *C*_AM_ is the Kullback-Leibler divergence (AM divergence).

The *r*_*π*_^*x*^(*k*) in *C*_AM_(*v*, *r*) is a distribution from the teacher model.

Additionally, *C*_AM_(*r*_*π*_^*x*^, *r*_*π*_) = *B*(*r*_*π*_^*x*^, *r*_*π*_) − *B*(*r*_*π*_^*x*^), where *B*(*r*_*π*_^*x*^) is a constant entropy. Therefore, Equation (4) can be reframed as the following equation.

(6) $$\begin{array}{c} m_{\text{AC}}=\left(1-\beta \right)B\left(n,r\right)+\beta \left(C_{\text{AM}}\left(r_{\pi }^{x},r_{\pi }\right)+B\left(r_{\pi }^{x},r_{\pi }\right)\right)=\left(1-\beta \right)B\left(n,r\right)+\left(\beta B\left(r_{\pi }^{x},r_{\pi }\right)\right). \end{array}$$

Setting the temperature *π* = 1 and $m_{\text{AC}}=B\left({\tilde{n}}^{x},r\right)$, where ${\tilde{n}}^{x}$ is as follows:

(7) $$\begin{array}{c} {\tilde{n}}^{x}\left(a\right)=\left(1-\beta \right)n\left(a\right)+\beta r^{x}\left(a\right). \end{array}$$

### 3.3. Reverse Knowledge Distillation in Theory

Unlike normal KD, Re-KD takes teachers' accuracy as the baseline accuracy, which is much advanced than normal KD. For example, in various cases, Re-KD exceeds the normal KD. The basis of this concept is that the teacher becomes the student and the student becomes the teacher. Using Re-KD in the BACH dataset for cancer histopathology biopsy images, we found that Re-KD produces better results.

### 3.4. Bilateral Knowledge Distillation in Theory

For conventional knowledge, distillation of the loss function is mathematically defined as follows:

(8) $$\begin{array}{c} M_{\text{WAC}}=\delta \left(j,j^{\prime }\right)+\underset{h\varepsilon H}{\sum }\eta_{h}\rho_{h}\left(E_{h}^{S},E_{h}^{X}\right), \end{array}$$

where *δ*(*j*, *j*′) represents loss of task-specific nature, *j* is the ground truth, transformed output of the student layer is represented as *E*_*h*_^*S*^, transformed output of the teacher network is represented as *E*_*h*_^*X*^, note that this transformed module is produced from *m*-th module, *η*_*h*_ is a tunable balance factor which balances the unlike losses, *ρ*_*h*_(·, ·) is the *m*-th distillation loss to reduce the difference between *E*_*h*_^*S*^ and *E*_*h*_^*X*^.

Consider *kf* ∈ {0, 1} to be a Bernoulli random variable, and *f* is the *f*-th hybrid block in the hybrid network. Assuming (*kf* = 1) as the student path selected and when the teacher path is chosen, it is assumed as (*kf* = 0). Suppose *B*_*f*_ represents the input and *B*_*f*+1_ depicts the output of the *f*-th hybrid block; hence, the yield *f*-th hybrid block can be represented as follows:

(9) $$\begin{array}{c} B_{f+1}=k_{f}I_{f}^{S}\left(B_{f}\right)+\left(1-\beta_{f}\right)I_{f}^{X}\left(B_{f}\right). \end{array}$$

Here, *I*_*f*_^*S*^(·) is the functional representation of the student block and *I*_*f*_^*X*^(·) is the functional representation of the teacher block.

Taking the value of *β*_*f*_ to be 1, Equation (2) takes the following form:

(10) $$\begin{array}{c} B_{f+1}=I_{f}^{X}\left(B_{f}\right). \end{array}$$

This simply means the hybrid block reduces to the original student block. Whereas if we consider *β*_*f*_ = 0, Equation (2) can be formulated as follows:

(11) $$\begin{array}{c} B_{f+1}=I_{f}^{X}\left(B_{f}\right). \end{array}$$

Now suppose *δ*(., .) is the task-specific loss, *j* represents the ground fact ${\tilde{j}}_{y}$ denoting the predicted result of the hybrid network, and *d*_*y*_ is the hybrid network, its optimized loss function can be written as follows:

(12) $$\begin{array}{c} d_{y}=\delta \left(j,{\tilde{j}}_{y}\right). \end{array}$$

As per Figure 2 and Algorithm 1, we propose a bilateral knowledge distillation regime. In phase 1, the more complex teacher model, the ResNeXt29, is used as a teacher model to train the lightweight MobileNetV2. In step 2, the teacher and the student are reversed just being interactive and exchanging knowledge. It is already shown in the literature that the teacher and students can distil knowledge to each other. In this novel approach, phase 2 comes into a picture, where the learnings of the teacher and student are fed back to each other and improved accuracy at each phase. We have stopped in phase 3 where knowledge distillation through MobileNetV2 has produced state-of-the-art accuracy as discussed in our results. This process can be iterated over several phases until we get the desired accuracy and depending on the computational resources available. The idea is further illustrated in Figure 3 with a schematic description.

## 4. Results

### 4.1. Experimental Setup

For our experiments, we use two well-known transfer learning networks in the ImageNet dataset, ResNeXt29 and MobileNetV2 pretrained models. BACH 2018 dataset of breast histopathology images was trained on those networks for the training of histopathology images. PyTorch (build 1.9.0) with CUDA 10.2 platform was used for the experiments.

### 4.2. Baseline Teacher Training

Our baseline trainer training on ResNeXt29 (8 × 64 d with 34.53 M parameters) and MobileNetV2 (including the preliminary completely convolution layer with 32 filters, accompanied by the way of 19 residual bottleneck layers) indicates that the validation accuracy for ResNeXt29 is as excessive as 75 percent wherein as that of MobileNetV2 is 60.71 percent as shown in Figures 4 and 5.

### 4.3. Tuning Hyperparameters

Several hyperparameters were tuned as follows: Optimizer: SGD, momentum=0.9, weight_decay=5e-4, Learning Rate scheduler: learning rate warm up, Defined phase as n: 3, Define epochs as e: 200, “alpha”: 0.95, “temperature”: 20, “learning_rate”: 0.1, “batch_size”: 8, “dropout_rate”: 0.5, “save_summary_steps”: 100, “num_workers”: 4.

### 4.4. Normal Knowledge Distillation Results

Since ResNeXt29 gave us higher accuracy in validation, we proceed by taking it as a teacher network and taking MobileNetV2 as the lighter student network. As per literature, we confirmed that the teacher model was able to distil the lightweight student model. However, since histological images are computationally complex, the results were no more than 60.71 percent on the validation set. The loss was considerable. The normal KD results are shown in Figure 6.

### 4.5. Reverse Knowledge Distillation Results

Again, we reversed the teacher and student networks to validate the reverse knowledge distillation on the given set of histological images. As such, MobileNetV2 now becomes the teacher and ResNeXt29 becomes the student. The results were improved as we got a validation accuracy of 65.58 percent. The results which are obtained through these experiments are shown in Figure 7.

### 4.6. Bilateral Knowledge Distillation Results

From the results of the above two experiments, we infer that the normal KD or the reverse KD is not sufficient to give us the best result for computationally complex histological images. Our proposed method of bilateral knowledge distillation, which works on the notion of both teacher and student, interactively learns from each other and thereby improves each other's accuracy. After three phases of interactive learning and exchanging information between teachers and the student, the MobileNetV2 reaches 96.3 percent accuracy on a validation set, which we claim as a state-of-the-art result for histological images of the breast. Results of training and validation using bilateral knowledge distillation are shown in Figure 8.

## 5. Discussion of Results

In bilateral cognitive distillation, we found that students and teachers interact with each other. In noninteractive cognitive distillation such as traditional cognitive distillation, the teacher network sets only one goal to mimic the student network, ignoring the communication of the student network. However, since the characteristic transformation potential of the student network is much lower than that of the teacher, it is impossible to mimic the exact knowledge that the teacher has transferred to it. Therefore, there is a difference between the knowledge taken by the student and the knowledge transferred by the teacher, which limits KD performance. In interactive, bilateral cognitive distillation, the student takes action based on the problem they are facing, then the teacher gives feedback based on the student's actions, and finally, the student takes action according to the teacher feedback. In particular, we propose that the teacher and students be interactive and that knowledge be transferred from teacher to student and from student to student to teacher until the student who assesses the classes reaches the allowable accuracy. We used two pretrained models trained on ImageNet datasets for our baseline training, namely, ResNeXt29 and MobileNetV2, for validation of theories of knowledge distillation on breast histological images. The histology biopsy images are too complex and have a similar colour combination when viewed under a microscope after staining. As such even with robust networks like ResNeXt29 and MobileNetV2, the base line accuracies were limited. In normal KD, due to higher validation accuracy, ResNeXt29, the more complex model has been chosen as the teacher network and the simple MobileNetV2 as the corresponding student network and the teacher and student networks were reversed for Re-KD. After three phases of interactive learning and exchanging information among teacher and the student, the MobileNetV2 reaches 96.3 percent accuracy on validation set which we claim as a state-of-the-art result for histological images of the breast. The limited accuracy obtained through these conventional methods prompted us to run the experiment with bilateral-interactive KD. As knowledge distillation is nothing but a regularization technique, the student network is seldom overfitted and it can backpropagate the errors. Therefore, there is a constant feedforward and backpropagation across the different phases of the bilateral KD model. In each phase, the labels are smoothed with regularization and hence the forth accuracy improves with each phase. All the results we discussed can be summarized in Table 2 below. We also conclude that with the increase of temperature, the distribution of soft targets in the teacher network mimics the uniform distribution of label smoothing. The other important observation in this experiment is the fact that bilateral KD does not need additional distillation losses and is in accordance with the conventional KD method.

## 6. Conclusion

In this paper, we have discussed the results obtained in two baseline papers on knowledge distillation and interactive knowledge distillation. We proposed a novel method called bilateral knowledge distillation on breast histological images. In our approach, we took ResNeXt29 and MobileNetV2 as the baseline pretrained models. The phenomenon that knowledge distillation is nothing but a label smoothing regularization technique was established yet again through the experiments conducted on histological image dataset of the breast. Additionally, the idea that label smoothing regularization is an ad hoc KD is reestablished. The interactive bilateral KD model which we proposed conforms to the fact that the teacher and student blocks interact with each other and is capable of transferring knowledge to each other through the correspondence being established and that this correspondence improves the accuracy in each subsequent phase. In normal KD, due to higher validation accuracy ResNeXt29, being the more complex model has been chosen as the teacher network and the simple MobileNetV2 as the corresponding student network and the teacher and the student networks were reversed for Re-KD. The limited accuracy obtained through these conventional methods prompted us to run the experiment with bilateral-interactive KD. The choice of transfer learning architecture was being validated by a baseline training. The result of bilateral KD is that the MobileNetV2 network produced excellent accuracy in phase 3 of the validation. Being a lightweight model, MobileNetV2 architecture will support deployment of the model in mobile applications also. The challenges of working with large-sized histological images and computational complexity can thus be avoided. This approach produces state-of-the-art results with an accuracy of 96.3 percent. It will also boost the performance of the student model on complex and diverse cancer cell images. Moreover, the model does not rely on copying the teacher behaviour, but rather it can utilize the feature transformational ability of the teacher. Going forward, we believe that this paper will help researchers to work with histological data of other cancers as well.

## Figures and Tables

**Figure 1:** The labelled images of each type of cell used in classification.

**Figure 2:** The proposed framework of knowledge distillation.

**Figure 3:** Schematic flow diagram of bilateral KD as used in this paper.

**Figure 4:** Train and test set accuracy of MobileNetV2.

**Figure 5:** Train and test set accuracy of ResNeXt29.

**Figure 6:** Normal knowledge distillation results.

**Figure 7:** Reverse knowledge distillation result.

**Figure 8:** Results of training and validation using bilateral knowledge distillation.

**Algorithm 1:** Bilateral knowledge distillation (base training: ResNeXt29 for e epochs).

**Table 1:** Specifications of microscopy images.

*S* no.	Parameter	Details
1	Colour model	Red, green, blue
2	Size	2048(*W*) × 1536(*L*) in pixels
3	Pixel scale	0.42 *μ*m × 0.42 *μ*m
4	Retention area: 10-20 MB (approx.)	10-20 MB (approx.)

**Table 2:** Results of all experiments performed.

Experiment performed	Model	Validation accuracy
Baseline teacher training	ResNeXt29	75%
	MobileNetV2	60.71%

Normal KD	ResNeXt29 teacher	60.71%
	MobileNetV2 student	

Reverse KD	MobileNetV2 teacher	65.58%
	ResNeXt29 student	

Bilateral KD	Phase 1+phase 2+phase 3	96.3%

## Data Availability

Data will be made available on request.
